This article has been retracted.

# Role of scientific and technological innovations on industrial upgradation in China: A spatial econometric analysis

**DOI:** 10.1371/journal.pone.0304344

**Published:** 2024-05-30

**Authors:** Yankun Liu, Ghulam Rasool Madni

**Affiliations:** 1 School of Urban Economics, Lanzhou City University, Lanzhou, China; 2 Department of Economics, Division of Management and Administrative Science, University of Education, Lahore, Pakistan; National University of Singapore, SINGAPORE

## Abstract

China is in a phase of high-quality development, where scientific and technological innovations are serving as the primary driving force for its development strategy. This emphasis on innovations is expected to fuel the upgrading of the industrial structure. This study investigates the role of scientific and technological innovations in industrial upgradation in China using spatial econometric analysis. Leveraging the data of 31 provinces of China from 2005 to 2022, we employed a spatial Durbin model to determine the spatial spillover effects of scientific and technological innovations on industrial upgradation. Our findings reveal the significant positive spatial spillover effects, indicating that provinces with higher levels of scientific and technological innovations tend to experience greater industrial upgradation, which in turn contributes to regional economic development. Furthermore, the findings suggest a strong spatial correlation between innovation and the upgrading of industrial structures, indicating that regional innovations have the potential to drive China’s industrial upgradation. These results underscore the critical role of scientific and technological innovations in promoting industrial upgradation and regional development in China.

## 1. Introduction

Upgrading and transformation of the industrial sector refer to the process of improving the quality, efficiency, and competitiveness of industries through technological advancements, organizational changes, and innovation. It involves shifting from traditional, low-value-added activities to more advanced, high-value-added activities. Upgrading and transformation of the industrial sector is essential for enhancing competitiveness, fostering innovation, and ensuring sustainable growth. This process requires careful planning, investment in research and development, adoption of new technologies, and support for workforce training [1]. China’s supply-side reform represents a fundamental shift towards the upgradation of its industry. This reform is a crucial step in enhancing the efficiency of the supply chain, boosting consumption growth, and driving overall economic expansion. Technological innovation plays a pivotal role in this transformation, serving as a key driver for upgrading industrial structures and propelling economic development forward [2]. At the strategic level, the Chinese government places significant emphasis on technology, particularly in research and development (R&D) and innovations, as crucial elements in the process of industrial upgradation. This shift necessitates continuous optimization and upgrading of the economic structure [3].

Technological and scientific innovations describe the development and implementation of new or significantly improved products, processes, services, or methods. These innovations often result from scientific discoveries, technological advancements, or creative ideas that lead to practical applications with economic or social value. Technological and scientific innovations play a crucial role in driving industrial upgradation because innovations lead to the development of new products, processes, and technologies, which can enhance the competitiveness of industries in both domestic and global markets [4]. Innovative technologies and processes often result in increased productivity, allowing industries to produce more with the same or fewer resources. It can lead to the improvement of product quality, helping industries meet higher standards and customer expectations [5]. Innovative technologies and processes may help the industrial sector to use resources more efficiently, reducing waste and environmental impact. Overall, innovations are essential for industrial upgradation as they drive efficiency, competitiveness, and sustainability, leading to the economic growth and development of a country [6].

Existing research on the relationship between innovations and industrial upgradation can be categorized into two main directions: single research and interactive research. Rostow [7] argued that the development of technology and industrial structure are interactive and mutually reinforcing during economic growth. The evolution of modern technology has a significant role in the transformation of traditional agriculture into industrialization. Concurrently, the continuous industrialization and emergence of new industries have propelled the reform and innovation of technology to meet the demands of industrial upgradation. Porter [8] identified technological innovation as the most critical factor in promoting industrial restructuring. Greunz [9] investigated the external effects of innovation growth using the MAR model, revealing that knowledge spillovers and patent application activities primarily occur within the core industry, with high-tech innovation dependent on the diversity of industrial structure. Iammarino and McCann [10] theoretically analyzed the relationship between the location development model, technological innovation process, and industrial agglomeration and upgrading. They suggested that geographical location, information technology, and knowledge spillover promote industrial agglomeration and continuous optimization and upgradation within regions, facilitating knowledge dissemination and technology creation. Bogliacino et al. [11] established a regression model based on manufacturing and service industries in European countries, finding that technological change, based on knowledge creation, product innovation, and new market development, is a key driver of differences in industrial structure changes across countries. Antonelli [12] compared the interaction between innovation and industry to two aspects of the same coin, suggesting that the speed and direction of technological change depend on the specific characteristics and trends of the industry and economic structure at each time point. Coad et al. [13] emphasized that enterprise R&D, innovation, and technological development are crucial drivers of job creation, welfare, and economic growth, marking changes in countries’ industrial structures. Using the C-D production function, Wakelin [14] demonstrated that R&D investment significantly promotes improvements in industrial production efficiency. Peneder [15] asserted that technological progress promotes industrial structure upgrading by enhancing factor production efficiency, deepening the social division of labor, and efficiently allocating resources, identifying it as a crucial factor in promoting industrial structure upgrading.

Several scholars have delved into the mechanisms through which technological innovations impact the upgrading of industry, focusing on aspects such as the labor force, industrial competitive advantage, and technological differentiation. Stoneman [16] posited that science and technology development influences the distribution of the workforce, facilitating the transition of labor from primary to higher value-added industries, thereby propelling industrial upgrading. Porter [17] also argued that industries gain competitive advantage through the continuous iteration of innovative technologies, thus driving internal structural upgrades, a concept he related to his ’diamond model. Bogliacino et al. [11], drawing on the ’New Schumpeterian’ school theory, conducted an empirical analysis across six major European countries, demonstrating how technological innovation impacts national industrial structure levels. This research highlighted that varying levels of technological innovation result in different national industrial structures, underscoring the significant role of technological innovation in national industrial structure development.

Studying the role of innovations in industrial upgrading in China is crucial for several reasons. China’s economy is undergoing a transition from being driven by investment and exports to being driven by innovation and consumption. Understanding how innovations contribute to industrial upgrading can help sustain economic growth. China is seeking to upgrade its industries to higher value-added activities. Studying the role of technological innovations can provide insights into how industries can transform and remain competitive in the global market. Moreover, the Chinese government has implemented various policies to promote innovations and industrial upgradation. Research in this area can help to evaluate the effectiveness of these policies and inform future policy decisions. Based on the importance of the topic, this study investigates the link between technological innovations and industrial upgradation by conducting a spatial analysis of China’s provincial data. The goal is to understand the relationship between technological innovations and the upgradation of industry by applying spatial econometric analysis. The use of spatial econometrics allows to account for spatial dependencies among observations, which is crucial when analyzing regional or local economic phenomena like industrial upgradation. This approach goes beyond traditional econometric techniques by incorporating spatial effects into the model, which can provide more accurate and robust estimates. The Spatial Durbin Model also allows for the estimation of both direct and indirect effects of scientific and technological innovations on industrial upgradation. This model is well-suited for analyzing spatially correlated data and can provide insights into how innovations in one region may spill over to neighboring regions. This approach also addresses the endogeneity concerns by using instrumental variable techniques or other methods to deal with potential biases that could arise from the simultaneity of innovation and industrial upgradation.

The study focuses on analyzing the relationship between scientific and technological innovations and industrial upgradation in China from a spatial perspective. This means that it considers not only the direct effects of innovations but also how these effects might vary spatially and how innovations in one region may impact industrial upgradation in neighboring regions. Moreover, the use of spatial econometric analysis is a novel approach that allows the study to account for spatial dependencies and heterogeneity in the data. This approach goes beyond traditional econometric methods by explicitly modeling spatial relationships, which can provide more accurate and insightful results. While there have been studies on the role of innovations in industrial upgradation in general, focusing specifically on China adds novelty. China’s rapid industrialization and economic growth make it an interesting case study, and the findings of the study could have implications for other developing countries undergoing similar transitions. In addition, the study likely provides policy-relevant insights into how scientific and technological innovations can be leveraged to promote industrial upgradation in China. This could be of great interest to policymakers and industry stakeholders looking to drive economic development and innovation in the country.

Additionally, the study aims to assess the role of innovations in driving the upgradation of industrial structures. This research is highly relevant for identifying viable pathways for transforming economic growth drivers in the contemporary era, facilitating a seamless transition between new and traditional sources of economic vitality, and ensuring the maintenance of stable economic development.

## 2. Theoretical foundations

The theory of innovations encompasses various perspectives and frameworks that seek to understand how new ideas, products, processes, or technologies are developed, adopted, and diffused within society. One of the seminal works in this area is Schumpeter’s theory of economic development, which highlights the role of entrepreneurs in driving innovation and growth. Schumpeter’s theory posits that innovations are the primary driver of development, leading to the creation of new industries and the transformation of existing ones [18]. Schumpeter argued that innovations are driven by entrepreneurs who are willing to take risks and introduce new ideas into the market. One of the key concepts in Schumpeter’s theory is the idea of "creative destruction." While this process can lead to the decline or even destruction of established businesses, it also drives economic growth and progress by fostering competition and innovation. Another aspect of the theory of innovation is the concept of diffusion. It means the spread of new ideas, technologies, or practices within society. In addition to Schumpeter’s work, other theories of innovation have emerged that focus on different aspects of the innovation process.

The theory of industrial upgrading refers to the process by which industries improve their capabilities, technologies, and products to move up the value chain and become more competitive in the global market. Industrial upgrading is essential for economic development, as it allows countries to diversify their economies, increase productivity, and create higher value-added products and services [19]. There are several theories and frameworks that help explain the process of industrial upgrading. Product life cycle theory was proposed by Raymond Vernon in the 1960s, this theory suggests that products go through distinct stages of development, from introduction to growth, maturity, and decline. According to this theory, companies in developed countries initially innovate and introduce new products, but as products mature, production shifts to developing countries where costs are lower [20]. This process can lead to industrial upgrading in developing countries as they move from producing basic goods to more advanced products.

Global value chain theory, developed by Gereffi, Humphrey, and Sturgeon, emphasizes the importance of global value chains (GVCs) in shaping industrial upgrading. GVCs are the full range of activities involved in the production of goods and services, from design and production to marketing and distribution [21]. The theory suggests that participating in GVCs can help firms in developing countries acquire new technologies, skills, and knowledge, leading to industrial upgrading [22]. Industrial upgrading is often driven by learning and capability building within firms and industries. As firms gain experience in producing and exporting goods, they develop new skills, technologies, and organizational capabilities. This learning process can lead to the development of more advanced products and processes, enabling firms to move up the value chain [23]. Industrial upgrading is closely linked to innovation and technology transfer. Technology transfer, through foreign direct investment (FDI) or partnerships with multinational companies, can also facilitate industrial upgrading by providing access to new technologies and markets [24]. Industrial upgrading is often supported by government policies and institutions that promote innovation, investment, and trade. Governments can provide incentives for firms to invest in R&D, improve infrastructure, and enhance the business environment. Strong institutions, such as effective legal systems and intellectual property rights protection, are also crucial for fostering industrial upgrading [25].

Technological innovation influences the upgrading of industrial structures through several mechanisms. Technological innovation can lead to the development of new production processes and technologies that improve productivity [26]. Technological innovation often results in the development of higher-quality products. Improved product quality can help firms differentiate themselves from competitors and capture higher market shares [27]. Technological innovation can enable firms to diversify their product offerings. By introducing new and innovative products, firms can enter new markets and reduce their reliance on a single product or market segment [28]. Technological innovation can lead to efficiency gains and these efficiency gains can result in cost savings and improved customer satisfaction [29]. This can help firms differentiate themselves in the market and capture higher profits [30]. Overall, technological innovation is a key driver of industrial upgrading, enabling firms to improve productivity, enhance product quality, diversify their product offerings, achieve efficiency gains, and gain a competitive advantage in the market.

## 3. Methodology

### 3.1. Data and Variables

In this study, industrial upgradation is a dependent variable. It refers to the process of improving and modernizing industrial infrastructure, processes, technologies, and practices to enhance efficiency, productivity, quality, and competitiveness. Industries need to stay relevant, meet changing market demands, and remain competitive in the global economy [31]. The variable of industrial upgradation is computed by considering the ratio of labor productivity in each industry to the proportion of output value of various industries in the total value. The main independent variable is scientific and technological innovations which is measured by the number of patents application acceptance. Moreover, based on earlier literature and theoretical foundations [7–9, 15, 22, 28], “the control variables of the study are per capita GDP, the level of urbanization is measured by the proportion of urban population in total population, the degree of openness is proportion of the total import and export volume of the region in the GDP, informatization is Internet users in total population, government intervention represented by government financial expenditure/GDP, and FDI is percentage of GDP” [32]. Per capita GDP is a proxy for the overall economic development level of a region. Regions with higher per capita GDP are likely to have more resources and infrastructure to support technological innovations and industrial upgradation. By including per capita GDP as a control variable, the study can better isolate the effects of innovations on industrial upgradation, controlling for the level of economic development. Moreover, regions with higher per capita GDP may have greater demand for innovative products and services, which can drive technological innovations in industries. Including per capita GDP as a control variable helps to account for this demand-driven aspect of innovation.

It is argued that urban areas tend to have better infrastructure, including transportation networks, communication systems, and research facilities. Higher levels of urbanization can facilitate the adoption and implementation of technological innovations, which are crucial for industrial upgradation. Urban areas often have larger and more accessible markets, which can incentivize firms to innovate and upgrade their industrial processes to meet the demands of urban consumers. Including urbanization as a control variable helps to account for these market dynamics. Urban areas serve as hubs for innovation and knowledge spillovers, which can benefit neighboring regions. Including urbanization as a control variable helps to account for these spatial spillover effects and their impact on industrial upgradation.

Trade openness can facilitate the transfer of technology and knowledge between the regions. Regions that are more open to trade may have greater access to new technologies and innovative practices, which can stimulate industrial upgradation. It can increase market competition, incentivizing firms to innovate and upgrade their industrial processes to remain competitive in international markets. Including trade openness as a control variable helps to capture the effects of this competitive pressure on industrial upgradation.

Informatization reflects the degree to which digital technologies are integrated into various aspects of society and the economy. Regions that are more advanced in informatization are likely to have better infrastructure and capabilities to support technological innovations and industrial upgradation. Informatization levels can vary significantly between regions, leading to disparities in access to digital technologies and skills. Including informatization as a control variable helps to account for these regional differences and their potential impact on the relationship between innovations and industrial upgradation. Informatization enables the collection and analysis of large amounts of data, which can fuel data-driven innovation in industries such as healthcare, finance, and manufacturing.

Government intervention can have a significant impact on the level of scientific and technological innovations in an economy. Policies such as research grants, tax incentives, and technology subsidies can stimulate innovation and industrial upgradation. Government regulations can also influence the level of innovation and industrial upgradation in an economy. For example, regulations related to intellectual property rights (IPR), competition, and environmental standards can affect firms’ incentives to innovate. Governments often provide support to specific industries or sectors through subsidies, grants, and other forms of assistance. This support can influence the level of innovation and industrial upgradation in these industries. Government intervention can also vary between regions, leading to disparities in the level of innovation and industrial upgradation.

FDI can facilitate the transfer of technology and knowledge from foreign firms to domestic firms, which can stimulate technological innovations and industrial upgradation. FDI can provide domestic firms with access to foreign capital and markets, which can help them invest in R&D and innovation. FDI can increase competition in domestic markets, leading to efficiency improvements and innovation incentives for domestic firms. Additionally, FDI can create spillover effects, where knowledge and technology transfer from foreign firms benefit domestic firms. FDI is often influenced by government policies, such as investment incentives and regulations. These policies can affect the level of FDI and its impact on industrial upgradation. FDI inflows can vary between regions, leading to disparities in the level of industrial upgradation.

The data of these variables is collected from the “China Statistical Yearbook” and “China Science and Technology Statistical Yearbook” for the period from 2005 to 2022 covering 31 provinces of China.

### 3.2. Model

Exploratory Spatial Data Analysis (ESDA) is a set of techniques used to analyze and visualize spatial data to uncover patterns, trends, and relationships that may exist in the data. ESDA is particularly useful for understanding the spatial distribution of variables and identifying spatial autocorrelation, which is the degree to which the values of a variable are correlated in space. It builds on the basic linear regression model but incorporates spatial dependencies among observations. Here are the key assumptions of the Spatial Durbin Model. The relationship between the dependent variable and the independent variables is assumed to be linear. The dependent variable is assumed to be spatially autocorrelated, meaning that the value of the dependent variable at one location is correlated with the values of the dependent variable at neighboring locations. This is captured by the spatial lag term, which is the weighted average of the dependent variable in neighboring locations. The error term is assumed to be spatially autocorrelated, meaning that the errors at one location are correlated with the errors at neighboring locations. The independent variables should not be perfectly correlated with each other. The spatial lag of the dependent variable should not be correlated with the error term. The error term should not be spatially autocorrelated. The errors should be independent and homoscedastic (have constant variance). The errors should be normally distributed. Violations of these assumptions can lead to biased and inconsistent parameter estimates, affecting the reliability of the model’s results. Global Moran’s I value describe the correlation across the sample area. The “GM’s I” test is specified as:

$$I=\frac{n\sum_{t=1}^{n}\sum_{j=1}^{n}Wij(Yi-\bar{Y})(Yj-Y)}{\sum_{t=1}^{n}\sum_{j=1}^{n}Wij\sum_{t=1}^{n}{\left(Yi-Y\right)}^{2}}$$

“The n shows the number of regions while Yi and Yj denote the observed value of region *i* and *j*. Wij represents the spatial weight matrix (SWM). The spatial weight matrix is a crucial component in spatial econometric analysis, and it defines the spatial relationships between different regions or spatial units and is used to capture the spatial dependencies in the data. There are several methods for constructing a spatial weight matrix, including Contiguity-Based Weights: This method defines spatial relationships based on contiguity or adjacency between spatial units. For example, a common approach is to use binary weights, where neighboring units are assigned a weight of 1 and non-neighboring units are assigned a weight of 0. Alternatively, contiguity-based weights can be based on the distance between units, with closer units assigned higher weights. The value of GM’s I test lies between -1 to 1. The value near to 1 reveals the strong positive spatial correlation while value closer to -1 highlights the strong negative spatial correlation. The Z value is applied to find the significance level of GM’s I test following the standard normal distribution” [33]. The derivation is as follows;

$$Z_{I}=\frac{I-E[I]}{\sqrt{Var[I]}}$$

In above equation, E[I] is expected value while Var [I] shows the variance of GM’s I. The “spatial autocorrelation model” (SAC), “spatial error model” (SEM), and “spatial autoregressive model” (SAR) are different categories of spatial econometrics model. The SAC model shows the spatial dependence between error term and dependent variable. The specification of SAC model is as follows;

$$z=\alpha W_{1z}+\beta i_{n}+ϒB+\mu$$

The spatial dependence of error term is determined through SEM model and specification of SEM model is as follows;

$$z=\beta i_{n}+ϒB+\mu$$

The spatial dependence in explained variable is determined through SAR model. The matrix from of SAR model is represented as:

$$z=\alpha Wz+\beta i_{n}+ϒB+\epsilon$$

The spatial dependence of lagged values of independent and dependent variables are estimated through “spatial Durbin model” (SDM) and specification of SDM is given as follows;

$$z=\alpha Wz+\beta i_{n}+ϒB+\varphi WB+\epsilon$$

The econometric model for estimation is as following:

$$IDU=a+\alpha WIDU+{ϒ}_{1}PTA+{ϒ}_{2}PCY+{ϒ}_{3}UBZ+{ϒ}_{4}INF+{ϒ}_{5}OPS+{ϒ}_{6}GOV+{ϒ}_{7}FDI+\varphi_{1}WPTA+\varphi_{2}WPCY+\varphi_{3}WUBZ+\varphi_{4}WINF+\varphi_{5}WOPS+\varphi_{6}GOV+\varphi_{7}FDI+\epsilon$$

where IDU is industrial upgradation and represents the dependent variable, while exogenous variables are scientific and technological innovations (PTA), PCY is per capita GDP, UBZ is urbanization, INF is informatization, OPS is openness, GOV is government intervention, and FDI is foreign direct investment. The details of each variable is already given in methodology.

## 4. Empirical findings

The Table 1 shows the findings of GM’s I index for industrial upgradation and innovations. The Z values are highly significant and positive, revealing the presence of spatial dependence.

**Table 1:** GM’s I of industrial upgradation.

**Years**	**2005**	**2006**	**2007**	**2008**	**2009**	**2010**	**2011**	**2012**	**2013**
GM’s I	0.32	0.31	0.32	0.41	0.47	0.24	0.34	0.33	0.48
p value	0.01	0.02	0.01	0.03	0.00	0.01	0.02	0.01	0.03
z value	3.63	4.28	4.51	4.37	4.31	3.95	3.87	4.07	5.17
**Years**	**2014**	**2015**	**2016**	**2017**	**2018**	**2019**	**2020**	**2021**	**2022**
GM’s I	0.31	0.44	0.45	0.31	0.24	0.29	0.34	0.42	0.43
p value	0.02	0.01	0.03	0.04	0.01	0.00	0.02	0.00	0.01
z value	4.67	4.31	4.68	5.27	4.39	5.39	4.32	3.62	4.52
**GM’s I of Innovations**									
**Years**	**2005**	**2006**	**2007**	**2008**	**2009**	**2010**	**2011**	**2012**	**2013**
GM’s I	0.16	0.17	0.22	0.23	0.24	0.28	0.30	0.33	0.35
p value	0.01	0.02	0.01	0.03	0.01	0.01	0.02	0.01	0.03
z value	2.68	3.25	3.51	3.38	3.36	2.99	2.86	3.02	4.17
**Years**	**2014**	**2015**	**2016**	**2017**	**2018**	**2019**	**2020**	**2021**	**2022**
GM’s I	0.34	0.32	0.30	0.26	0.24	0.23	0.22	0.21	0.22
p value	0.02	0.01	0.03	0.04	0.01	0.00	0.02	0.00	0.01
z value	3.66	3.38	3.62	4.27	3.37	4.39	3.39	3.62	3.58

According to the calculation formula of the global Moran’s I index, we take the industrial structure upgrading and innovations as the observation value, and the geographic distance matrix as the spatial weight matrix, and calculated the global Moran’s I index value. Table 1 indicates a growing spatial spillover effect of innovations and industrial upgradation. The findings reveal a significant positive correlation between industrial structure upgrading and spatial dynamics, consistent over time. This suggests a divergence in industrial development among China’s regions, leading to the formation of diverse industrial models. These trends align closely with the evolving landscape of China’s economic development.

After assessing the spatial effects of industrial upgradation and innovations, a regression analysis was conducted. The results indicate that the Spatial Durbin Model (SDM) is particularly effective in illustrating the impacts of exogenous variables on the ecological footprint, as it achieved the highest adjusted R2 value and the lowest values of HQ, SC, and AIC. To ensure the robustness of the empirical findings, four spatial models were employed, including the "Queen-based contiguity weight matrix," "K nearest contiguity weights matrix," and "double rook contiguity weight matrix." The results of the LR test and goodness of fit demonstrate the superiority of the SDM over other spatial models. Details of the selected spatial weight matrix are presented in Table 2.

**Table 2:** Spatial models.

Variables	SEM	SAR	SAC	SDM
PTA	0.36**(0.017)	0.37**(0.012)	0.31** (0.016)	0.37**(0.012)
PCY	0.84*** (0.055)	0.83*** (0.075)	0.85*** (0.047)	0.076***(0.049)
UBZ	0.02**(0.019)	0.03***(0.022)	0.02**(0.021)	0.03***(0.019)
INF	0.33(0.076)	0.44(0.068)	0.32(0.059)	0.29(0.072)
OPS	0.015(0.003)	0.018(0.002)	0.010(0.001)	0.019(0.004)
GOV	-0.038**(0.005)	-0.049**(0.004)	-0.046**(0.005)	-0.048***(0.003)
FDI	0.016*(0.015)	0.013(0.012)	0.012**(0.013)	0.016**(0.014)
Constant	-1.79**(0.316)	-2.76**(0.412)	-3.31**(0.274)	-4.53**(0.641)
**Spatial Effect**				
α		0.057(0.049)	0.073(0.038)	0.183(0.071)
φ	0.47**(0.061)		0.487**(0.068)	
W*PTA				0.52**(0.029)
W*PCY				0.07**(0.857)
W*UBZ				0.92**(0.045)
W*INF				0.85(0.019)
W*OPS				0.02(0.016)
W*GOV				-0.01**(0.184)
W*FDI				0.014**(0.015)
**Model Fitness**				
F-statistics	479.351**	563.543*	476.255*	507.416*
p-value	0.002	0.003	0.001	0.002
R2	0.92	0.93	0.91	0.96
Adjusted R^2^	0.91	0.91	0.90	0.95
HQ	0.052	0.426	0.514	0.381
SC	0.058	0.546	0.627	0.341
AIC	0.051	0.435	0.542	0.353

Note: *, **, and *** show significance level at 1%, 5% and 10% respectively.

The empirical results from the spatial Durbin model indicate a positive relationship with the lagged endogenous variable, suggesting that an increase in industrial upgradation in neighboring regions also positively influences industrial upgradation in one’s state. Additionally, the remaining spatial lagged exogenous variables show significant relationships, except for W*INF and W*OPS. This suggests that scientific and technological innovations have a positive impact on industrial upgradation in China. The per capita GDP demonstrates a significant positive impact on industrial upgradation, showing that as the level of economic development improves, the industrial structure becomes more optimized. Urbanization is also found to optimize the regional industrial structure; however, China’s relatively low level of urbanization hinders further upgradation of the industry. Surprisingly, informatization and openness do not show significant effects on industrial upgradation. Government intervention is found to inhibit industrial upgradation. Lastly, the spatial spillover effect of FDI on industrial upgradation between neighboring regions is positive.

## 5. Discussion

This study focused on exploring the impact of technological innovations on industrial upgradation and its spatial impact across the 31 provinces of China. It is found by empirical analysis that innovations have a significant positive impact on industrial upgradation. Innovations in technology have allowed Chinese industries to adopt advanced manufacturing processes, improve efficiency, and produce higher-quality products. This has helped industries move up the value chain and compete more effectively in global markets [34]. Innovation has led to the diversification of industries, with new sectors emerging and existing sectors upgrading. This diversification has reduced reliance on traditional industries and contributed to a more balanced and sustainable industrial structure [35, 36]. By investing in innovation, China has been able to improve the quality and competitiveness of its products, making them more attractive to international markets. This has helped Chinese industries expand their presence globally and compete with other leading economies [37–40]. It is also found that innovations have a spatial impact across provinces in China, with some regions benefiting more than others. Provinces with strong innovation ecosystems have seen rapid industrial upgradation and economic growth [41]. Other regions, particularly in the western part of the country, have lagged but are gradually catching up through targeted government policies and investments in innovation [42]. The spatial impact of innovations across provinces highlights the importance of regional development strategies and targeted investments in fostering innovation-led industrial upgradation across the country [33, 43].

The empirical analysis reveals that GDP has a significant positive impact on industrial upgradation. High GDP growth has allowed to invest heavily in infrastructure development, such as transportation networks, energy facilities, and communication systems. This infrastructure development has supported the growth of industries and facilitated industrial upgradation [44]. Growing GDP has led to an increase in consumer demand for goods and services. This increased demand has driven industrial expansion and encouraged industries to upgrade their products and processes to meet consumer needs [45]. Higher GDP has enabled China to invest in R&D and technology adoption. This has led to technological advancements in various industries, driving industrial upgradation and competitiveness [46]. The impact of GDP growth on industrial upgradation has also spatial correlation. Provinces with higher GDP growth, such as those in the eastern coastal region, have experienced more rapid industrial upgradation due to greater access to resources, markets, and infrastructure. In contrast, provinces in the western and central regions have seen slower industrial upgradation but are catching up as government policies and investments are directed towards promoting balanced regional development [47].

It is also found that urbanization in China has a positive impact on industrial upgradation. Urbanization has led to a significant increase in urban population in China. This has created a large and growing market for goods and services, driving demand for more advanced and high-quality products. As a result, industries have been incentivized to upgrade their products and processes to meet the needs of urban consumers [48]. Urbanization has spurred the development of urban infrastructure, including transportation networks, utilities, and communication systems. This infrastructure development has supported the growth of industries and facilitated industrial upgradation by improving access to markets, suppliers, and resources [49]. Urbanization has attracted rural residents and this led to an increase in urban labor force, providing industries with a larger pool of skilled workers. The availability of skilled labor has enabled industries to adopt more advanced technologies and production methods, leading to industrial upgradation [50]. Urbanization has led to the formation of industrial clusters in cities, where related industries and businesses concentrate in a specific geographic area. These clusters promote collaboration, knowledge sharing, and innovation among firms, leading to industrial upgradation and the development of new industries [45]. Urban areas tend to have a more developed innovation ecosystem, with research institutions, universities, and technology parks. This ecosystem fosters innovation and technology transfer, supporting industrial upgradation [51]. The empirical analysis highlights that urbanization in one area also has a spatial impact in neighboring regions.

The impact of informatization and openness on industrial upgradation in China has been perceived as relatively insignificant. While China has made significant strides in informatization, there are some challenges and these challenges can limit the extent to which informatization contributes to industrial upgradation. China’s approach to openness has often prioritized attracting foreign investment and expanding exports, sometimes at the expense of focusing on the quality and innovation of domestic industries [52, 53]. This focus on quantity over quality can limit the impact of openness on industrial upgradation. China’s openness has led to increased reliance on foreign technology and equipment, particularly in high-tech industries. This dependency can hinder domestic innovation and limit the ability of Chinese industries to upgrade [44, 54, 55].

Government interference has a negative impact on industrial upgradation in China. Government interference, such as subsidies, preferential policies, and regulations, can distort market signals and hinder the efficient allocation of resources. This can lead to the misallocation of capital and resources, hindering industrial upgradation [31]. Government policies that protect domestic industries from foreign competition can reduce incentives for industries to upgrade and innovate. This can lead to complacency and a lack of competitiveness in the long run [33]. Government interference can lead to inefficient resource allocation, with resources being directed towards politically favored industries or projects rather than those that would benefit most from upgrading. This can result in a misallocation of resources and hinder industrial upgradation.

FDI has facilitated the transfer of advanced technologies, management practices, and know-how to Chinese industries. This has helped domestic firms upgrade their technologies and improve their production processes. FDI has provided Chinese industries with access to new markets and distribution networks [33, 56]. This has enabled them to expand their reach and increase their competitiveness. FDI has brought in significant capital investment, which has helped Chinese industries modernize their facilities, upgrade their equipment, and improve their infrastructure. FDI has increased competition in the Chinese market, forcing domestic industries to become more efficient and innovative to remain competitive [49, 57]. This competitive pressure has driven industrial upgradation and technological advancement. FDI has integrated Chinese industries into global value chains, allowing them to benefit from international trade and investment. This has helped Chinese industries become more globally competitive and has facilitated industrial upgradation.

## 6. Conclusions

Based on an analysis of China’s provincial data from 2005 to 2022, this study employed the spatial econometric model to find the relationship between innovations and industrial upgradation in China. The findings indicate several key points: First, using exploratory spatial data analysis, the study reveals a significant positive spatial correlation between industrial upgradation and innovations. Secondly, a spatial econometric model allows for an empirical investigation into the impact of regional innovations on industrial upgradation. The results confirm that regional innovation contributes to China’s industrial upgrading and enhances its overall innovation capacity. Additionally, the study highlights the importance of spatial spillover effects in influencing China’s industrial upgrading. These findings offer valuable insights for China’s future industrial development, emphasizing the need to increase investment in innovation and shift towards an innovation-driven economic model.

### 6.1. Implications

The implications of the study are significant for policymakers, businesses, and researchers. The study underscores the importance of policies that promote scientific and technological innovations to drive industrial upgradation in China. Policymakers can design and implement targeted policies that incentivize innovation and support industries in upgrading their technologies and processes. The study highlights the spatial dimension of industrial upgradation in China, indicating that innovation capabilities and industrial upgrading are closely linked across regions. Policymakers should prioritize regional development strategies that focus on enhancing innovation capabilities and promoting industrial upgradation in less developed regions. Businesses should develop strategies that leverage scientific and technological innovations to improve their products, processes, and market position. Moreover, based on the findings of this study, several practical policy recommendations are suggested to promote industrial upgradation through scientific and technological innovations. The government may increase the funding for R&D activities to encourage scientific and technological innovations. This can be done through government grants, tax incentives, and partnerships with universities and research institutions. Facilitate the transfer of technology from research institutions and universities to industries. This can be achieved through technology parks, incubators, and partnerships with foreign technology firms. Provide financial and technical support to SMEs to help them adopt and implement new technologies. This can include grants, low-interest loans, and training programs. Create innovation clusters or hubs where companies, research institutions, and government agencies can collaborate and exchange ideas. This can help stimulate innovation and promote industrial upgradation. Invest in education and skills development programs to ensure that the workforce has the necessary skills to support technological innovation and industrial upgradation. Improve infrastructure, such as transportation and communication networks, to support the diffusion of technology and facilitate collaboration between regions. Implement policies that promote balanced regional development, ensuring that the benefits of technological innovation and industrial upgradation are spread across different regions of China. These policy recommendations are based on the premise that scientific and technological innovations are key drivers of industrial upgradation and economic growth. Implementing these recommendations can help China to enhance its innovation capabilities and competitiveness in the global economy.

### 6.2. Limitations

This study has some limitations also that should be considered for future research. The study focused on the provincial level, which may not capture the full complexity of industrial upgradation in China. Industrial dynamics can vary significantly within provinces, and a more granular analysis at the city or district level could provide additional insights. Economic conditions and policy environments evolve from time to time so this factor may be considered for future studies. While the study provides insights into the role of innovation in industrial upgradation, it may not provide specific policies for a specific industrial sector. There are also some potential biases or constraints associated with the methodology and data used in this study. If the model does not properly account for spatial autocorrelation in the data, it can lead to biased parameter estimates. This bias occurs when the values of the dependent variable in one location are correlated with the values in neighboring locations, and this correlation is not captured in the model. Endogeneity occurs when the explanatory variables are correlated with the error term. In this context, it could happen if there are unobserved factors that affect both scientific and technological innovations and industrial upgradation. Failure to address endogeneity can lead to biased estimates of the impact of innovations on industrial upgradation. If important variables that are related to both innovations and industrial upgradation are omitted from the model, it can lead to biased estimates. For example, factors like government policies, market conditions, or cultural factors could influence both innovations and industrial upgradation. Establishing causality between scientific and technological innovations and industrial upgradation can be challenging. While spatial econometric models can help explore these relationships, they cannot establish causality definitively.
